This article has been retracted.

# Postoperative Effect Observation and Clinical Study of Dahuang Zhechong Pills from *Jingui Yaolue* in Treating Patients with Early-to-Mid Prostate Cancer Undergoing Radical Resection

**DOI:** 10.1155/2022/2998825

**Published:** 2022-04-27

**Authors:** Shizhao Hou, Chengguo Bin

**Affiliations:** ^1^Doctoral Student in Guangzhou University of Traditional Chinese Medicine, Emergency Department, Second Clinical Medicine of Guangzhou University of Traditional Chinese Medicine, Guangzhou City 510370, Guangdong Province, China; ^2^Department of Traditional Chinese Medicine, Dazu Hospital Affiliated to Chongqing Medical University, Chongqing City 402360, China

## Abstract

**Objective:**

To explore the effect of applying Dahuang Zhechong pills (DHZCP) from *Jingui Yaolue* to patients with early-to-mid prostate cancer undergoing radical resection and carry out a theoretical clinical study of traditional Chinese medicine (TCM) to verify the effect of DHZCP formula under the guidance of TCM theory.

**Methods:**

The clinical data of 98 patients with early-to-mid prostate cancer undergoing radical resection treated in our hospital (July 2014 to July 2016) were selected for the retrospective analysis, and the patients were divided into group A (*n* = 49, routine hormonal therapy) and group B (*n* = 49, routine hormonal therapy plus DHZCP) according to the double blind method, so as to compare the trauma symptoms, cancer recurrence rate, etc., after treatment between the two groups.

**Results:**

Compared with group A, group B obtained significantly higher total effective rate of complication treatment at different time points (*P* < 0.05), significantly lower mean HAMA score after treatment (*P* < 0.05), and significantly lower total recurrence rate (*P* < 0.05). The “congestion” theory in *Chapter VI On Pulse, Symptom Complex and Treatment of Arthralgia Due to Stagnation of Blood and Consumptive Diseases of Jingui Yaolue* was the theoretical basis for postoperative effect observation of DHZCP in treating prostate cancer. Combining with the onset theory of congestion, personally, the author believed that cancer is caused by congestion disease formed by the extravasated blood in the human body, and with the passing of time, the intermingled deficiency, blood stasis, and toxicity lead to the qualitative change of endogenous cancer toxicity and develop into consumptive congestion disease, making it the core pathogenesis of cancer. And DHZCP had good preventive and treatment effect.

**Conclusion:**

DHZCP is an effective drug for improving postoperative complications of early-to-mid prostate cancer, reducing the biological recurrence rate and clinical recurrence rate, and improving mental status. The formula treats both deficiency and excess, combines tonification with purgation, and dispels exogenous pathogen without damaging body resistance, which is a profound formula based on TCM theory to treat “congestion,” “congestion disease,” and “consumptive congestion disease.” Using this theory to guide clinical syndrome differentiation and treatment and modifying the dosage and usage can play an important role in TCM preventive treatment of cancers, early, middle, and late treatment, and clinical prevention of other chronic diseases.

## 1. Introduction

Prostate cancer is a common malignant neoplastic disease in elderly men [1], and globally, its incidence ranks second among all malignant tumors in men. Data from a US study survey [2] showed that prostate cancer incidence has surpassed that of lung cancer, and in Europe, approximately 2.6 million new cases of prostate cancer are diagnosed each year. The pathogenic mechanism of prostate cancer may be related to race, heredity, environment, food, smoking, sex hormone, etc. The disease is slowly progressive, with no specific manifestations in the early stage, and as the tumor grows gradually, it can invade into the urethra and bladder neck, often complicated by metastasis to bone and other routes and seriously threatening the life of patients [3,4]. Currently, radical prostatectomy is the first choice for treatment, with stable results. However, the complication incidence after radical prostatectomy is higher, with common postoperative complications including urinary tract pain, frequent micturition, and irritation sign of odynuria caused by anal, rectal, and perineal tenesmus, swelling and pain, abnormal defecation, urinary retention, urinary stenosis, and infection, which can seriously affect patients' recovery, mental status, and normal life [5]. Although conventional hormonal therapy after radical resection has shown good results for most patients in recent years, some patients inevitably experience biological recurrence and clinical recurrence, which eventually develop into metastatic castration-resistant prostate cancer. With the diversity of treatment modes, traditional Chinese medicine (TCM) can promote the improvement of patients' postoperative urination function and quality of life (QOL) [6,7] and is affirmed in the adjuvant and preventive treatment of cancer. The formula of Dahuang Zhezhong pills (DHZCP) is from *Jingui Yaolue* complied by Zhang Zhongjing, the medical sage at the end of the Eastern Han dynasty. With the in-depth study of DHZCP in recent years, it is found that the drug has merits in tumor inhibition and adjuvant treatment [8, 9]. However, no study has confirmed its efficacy in the adjuvant treatment after radical prostatectomy for early-to-mid prostate cancer. This study explored the effective mode of preventing and treating cancer with TCM by observing the efficacy of clinical application of DHZCP in improving the condition of patients undergoing radical prostatectomy and learning the scientific connotation of TCM theory of the formula by rethinking the classic TCM theories in *Huangdineijing* and *Jingui Yaolue*, so as to provide reference for the clinical application and study of DHZCP in TCM therapeutics and preventive treatment of disease.

## 2. Materials and Methods

### 2.1. General Data

The clinical data of 98 patients with early-to-mid prostate cancer undergoing radical prostatectomy treated in our hospital from July 2014 to July 2016 were selected for the retrospective analysis, all patients received relevant examinations, and the study met the World Medical Association Declaration of Helsinki (2013) [10].

### 2.2. Inclusion and Exclusion Criteria

Inclusion criteria: ① the patients were diagnosed with prostate cancer after pathological biopsy and had received radical prostatectomy; ② the patients were confirmed to have early-to-mid prostate cancer after pathological examination (Gleason score ≤ 7 points), and the manifestations of clinical symptoms were frequent micturition, urgent micturition, dysuresia, pelvic pain, etc.; ③ KPS score of the patients was > 70 points; ④ the patients had different degrees of trauma symptoms after surgery, including urinary irritation and anal, rectal, and perineal tenesmus, swelling, and pain. Exclusion criteria: ① the patients' tumor broke through capsule with distal metastasis; ② the patients were complicated with severe liver and kidney disorders or severe system disease; ③ the patients participated in other projects and studies; ④ the patients were confirmed to be allergic to the drug used in this study.

### 2.3. Methods

After surgery, routine hormonal therapy was performed to patients in group A. The patients orally took 50 mg of bicalutamide (NMPA approval no. H20113535; manufactured: Shanghai Fudan Forward Pharmaceuticals Co., Ltd.; specification: 50 mg *∗* 28 tablets) once daily and received 3.6 mg of goserelin (NMPA approval no. J20160052; manufactured: AstraZeneca PLC; specification: 3.6 mg × 1 bottle/box) via subcutaneous injection once every four weeks. Treatment and drug administration were maintained for half a year after t-PSA was below 0.2 ng/dl. During treatment, patients' various physical signs were monitored and their adverse drug reactions were observed. In case of poor efficacy or severe adverse drug reactions, detailed examinations were conducted and relevant preventive and treatment measures with western medicine were formulated.

After surgery, patients in group B received hormonal therapy and Dahuang Zhechong capsules, and the hormonal drugs and usage were the same as group A. Dahuang Zhechong capsules (manufactured: Jiangsu Ehai Pharmaceutical Corporation, Ltd.; NMPA approval no. Z20054026; specification: 0.4 g per capsule) were selected, and the composition and dose were based on the original formula of DHZCP from *Jingui Yaolue*, with twelve herbs (cooked rhubarb, Baikal skullcap root, liquorice root, peach seed, bitter apricot seed, Chinese peony, adhesive rehmannia dried root, dried lacquer, gadfly, a hundred leeches, white grub, and ground beetle) ground into powder and made into capsules. After surgery, the patients orally took 4 capsules each time and twice a day, patients at the early stage were administered for 3–6 months, and patients in the midterm were administered for 6–9 months. During treatment, patients' various physical signs were monitored, and their adverse drug reactions were observed. In case of poor efficacy or severe adverse drug reactions, detailed examinations were conducted, and corresponding controlling measures for the syndrome differentiation and treatment combining TCM with western medicine were formulated.

### 2.4. Efficacy Evaluation

The improvement of clinical complications (urinary irritation syndrome, difficult defecation, anal, rectal, and perineal tenesmus, swelling, and pain) in patients of the two groups after treatment was observed. ① Recovery criteria for urinary irritation syndrome [11]: after the end of follow-up, there were no white blood cells or red blood cells found in the urine by re-examination of routine urinalysis, and there were no bacteria in urine culture; ② recovery criteria for difficult defecation, anal, rectal, and perineal tenesmus, swelling, and pain [12]: normal frequency and time of defecation, smooth defecation, soft stools, and disappearance of abdominal distension, difficult defecation, anal, rectal, and perineal tenesmus, swelling, and pain.

The mental status of patients in the two groups was assessed by Hamilton Rating Scale for Anxiety (HAMA) [13], which is a common clinical scale used in the department of psychiatry, with the reliability coefficient (*r*) for total score of 0.93. The scale had 14 scoring items, and each item was rated by the 5-grade scoring method (on a scale of 0–4 points), with a total score of 56 points. Total score ≥29 points indicated severe anxiety, ≥ 21 points indicated obvious anxiety, ≥14 points indicated definite anxiety, ≥7 points indicated possible anxiety, and <7 points indicated no anxiety symptoms.

The occurrence of cancer of patients within 5 years was observed.

Biological recurrence: four ml of fasting venous blood was drawn from patients in the two groups in the morning and then put into the centrifugal tubes; the tubes were placed in 37°C for blood coagulation; after that, the blood was balanced and centrifuged to get the supernatant, i.e., the serum, which was extracted carefully and packaged for standby application. The total prostate-specific antigen (t-PSA) was measured by electrochemiluminescence assay. The normal range of t-PSA was 0–4 ng/dl, and if the measured t-PSA was over the normal value (0.2 ng/dl) twice, biological recurrence was confirmed. The numbers of cases with biological recurrence at different periods (0–30 months, 31–48 months, and 49–60 months) of the two groups were recorded.

Clinical recurrence: the patients were observed if they developed metastasis of cancer cells by other routes such as bone or lymph nodes during follow-up. Symptoms of bone metastasis of cancer cells: ① patients had local pain and radioactive and discharging pain at the metastatic sites; ② some patients had limited limb functional activity or presented with compression fracture and severe impairment of limb function, resulting in walking difficulties; ③ patients were prone to occur compression fracture, local joint stiffness, limitation of motion, etc; ④ t-PSA was obviously higher than 0.2 ng/dl. The numbers of cases with clinical recurrence at different periods (same as above) of the two groups were recorded.

### 2.5. Statistical Methods

In this study, the data were processed by the professional statistic software SPSS26.0, the picture drawing software was GraphPad Prism 7 (GraphPad Software, San Diego, USA), the enumeration data were examined by *X*^2^ test and expressed by [*n*(%)], the measurement data were examined by *t*-test and expressed by Mean ± SD, and differences were considered statistically significant at *P* < 0.05.

## 3. Results

### 3.1. Comparison of Clinical Data

No significant between-group differences in the clinical data such as mean age, KPS score, and pathological type were observed (*P* > 0.05), see Table 1.

### 3.2. Between-Group Comparison of Complication Treatment Effect at Different Periods

Compared with group A, the total effective rate of complication treatment at different periods was significantly higher in group B (*P* < 0.05), see Tables 2–4.

### 3.3. Between-Group Comparison of Patients' Mental Status after Treatment

The mean HAMA score after treatment was significantly lower in group B than in group A (*P* < 0.001), see Figure 1.

### 3.4. Between-Group Comparison of Recurrence Status during Follow-Up

The total recurrence rate of groups A and B was, respectively, 14.29% (7/49) and 2.04% (1/49), presenting significant difference between the two groups (*X*^2^ = 4.900 and *P* < 0.05), see Table 5.

## 4. Discussion

(I) With the improvement of living standards in recent years, people's dietary modes have changed greatly, resulting in prostate cancer prevalence increasing year by year [14]. The cause of prostate cancer remains unclear and may be related to multiple factors, such as race, heredity, environment, smoking, and hormone. Prostate cancer, which accounts for 11% of all male cancers and 9% of all male cancer deaths as reported in studies [15], has become one of the important causes of death in older men. The surgical treatment of prostate cancer has advanced greatly in recent years, with the implementation of radical prostatectomy becoming the first choice, because it can benefit patients, and the post-surgical 10-year survival rate can reach more than 90% [16, 17]. However, because prostate cancer may invade the urethra and bladder neck, a part of the functional urethra may be removed during the radical surgery, resulting in damage to related external sphincter, detrusor of bladder and vascular nerves, and impact on pelvic floor muscle, rectum and anal sphincter, and therefore, different degrees of urinary retention, urinary tract stenosis, frequent micturition, pain in urination, and other post-surgical urinary tract irritation signs will occur, which seriously affect patient's recovery progress, mental status, and prognosis [18]; meanwhile, how to reduce postoperative t-PSA biological recurrence and clinical recurrence, improve patient's QOL, and prolong patient's survival cycle is of great importance. In recent years, TCM has achieved great success in cancer prevention, adjuvant treatment, improving the QOL and prolonging life. The unique TCM theories and formulas can play an important role in the rehabilitation and prevention of recurrence after radical prostatectomy, which can regulate the overall syndrome of patients, has a rapid onset of treatment, high safety, and simple operation, and works better in treating postoperative complications, presenting significant application value [19, 20]. In addition, the view of cancer under the guidance of the idea of preventive treatment of disease in TCM is of great value in preventing cancer occurrence and progression. The study results showed that patients in group B, who received additional treatment with DHZCP, had significantly better efficacy in treating post-surgical complications than group A (*P* < 0.05), fully proving that DHZCP had significant efficacy in improving postoperative complications of radical prostatectomy. As for the postoperative recurrence, the 5-year recurrence rate of patients receiving DHZCP was only 2.04% (1/49), which was lower than those accepting the routine hormonal therapy (14.29%, 7/49), indicating that DHZCP could exert the effects of drastically removing blood stasis and various toxicities, warming yang and nourishing qi, promoting qi to activate blood, activating meridians and collaterals, and nourishing blood and promoting neovascularization [21,22], which can prevent the recurrence of tumor and work well in treating postoperative complications. Shortcomings of the study: limited by factors including time and conditions, the source of cases lacked diversity and the number of enrolled patients was small, which may affect the determination of the overall efficacy. On the basis of the current research, multicentered clinical studies with expanded sample size will be carried out in the future.

(II) TCM believes that the pathogenesis of cancer lies in the endogenous cancer toxicity caused by deficient vital qi and excessive pathogen, alteration of viscera, phlegm-dampness coagulation and aggregation, stagnation of qi and blood stasis, and internal binding of heat toxicity and that “deficiency, toxicity, and blood stasis” are the core causes of malignant tumors. TCM also points out that the reasons for postoperative recurrence of cancer are “remaining cancer toxicity” and “metastasis of cancer toxicity,” the main issues of cancer progression. From the onset and process of congestion, TCM holds that cancer is caused by congestion disease formed by the extravasated blood in the human body, and with the passing of time, the intermingled deficiency, blood stasis, and toxicity lead to the qualitative change of endogenous cancer toxicity and develop into consumptive congestion disease, which is the core pathogenesis of cancer and can occur in the whole body. Consumptive congestion disease can be either local lesion or systemic lesion and is prone to transmission. Its onset has the features of congestion and congestion disease, but is essentially different from the two [23]. DHZCP is from *Chapter VI On Pulse, Symptom Complex and Treatment of Arthralgia Due to Stagnation of Blood and Consumptive Diseases of Jingui Yaolue*, which is a classic formula to treat “consumptive congestion disease,” and has significant guidance meaning to the treatment of “congestion” and “congestion disease.” By applying the method of relaxing spleen-stomach and restoring vital energy, the formula works well in treating multiple diseases in clinic, presents obvious advantages in the treatment of cancer, and is of great application value in early prevention and adjuvant therapy of cancer, preventing recurrence, and promoting QOL and life cycle. The herbs in the formula have also shown considerable results in pharmacological and clinical research for the treatment of cancer. Implementing “reinforcement and elimination in combination” is an important rule in TCM to treat various neoplastic diseases, which is consistent with the strategies of regulating body immune function to resist diseases in modern medicine. DHZHP can activate the immune T cells in the human body and improve the immune function. Studies have shown [24] that tumor neovascularization is necessary for tumor growth and metastasis, and DHZCP can inhibit the proliferation of endothelial cells by interfering with the release of angiogenic factors; in addition, the formula is more advantageous in improving blood hyperviscosity status and inhibiting tumor cell invasion, and its efficacy has been confirmed in pancreatic cancer and gastric cancer [25]. This study addressed the treatment for patients after radical prostatectomy according to the treatment management of early-to-mid consumptive congestion disease, and the results also showed the promising future of the formula in the postoperative prophylaxis and treatment of prostate cancer.

The formula of DHZCP has unique advantages in principle, method, recipe, and medicines. Combining with the exposition of *Huangdineijing*, *Jingui Yaolue*, and famous experts to rethink the original meaning and dig the classic TCM theories and connotations has positive meaning to guide the clinical prevention and treatment of cancer. The following personal opinions were proposed for discussion with colleagues.

In *Chapter VI On Pulse, Symptom Complex and Treatment of Arthralgia Due to Stagnation of Blood and Consumptive Diseases of Jingui Yaolue*, it is pointed out that “extreme weakness due to five consumptions leads to emaciation and abdominal distension with no ability to eat, which is caused by improper diet, distress, improper drinking, excessive sexual intercourse, damage due to hunger, or overstrain injury, resulting in injured meridian, nutrient qi, and defensive qi, with the manifestations of congestion inside, squamous and dry skin, and darkness of the eye sockets. To relax spleen-stomach and restore vital energy, Dahuang Zhechong pills should be used as the main drug” [26]. It describes the cause, pathogenesis, and principle-method-recipe-medicines of “congestion,” “congestion disease,” and “consumptive congestion disease.”

(I) “Congestion” is the basis of the formation of congestion disease and consumptive congestion disease and the basic interpretation of the cause of the occurrence and progression of cancer. Congestion is a concept of disease, which first appeared in the sentence “with the manifestations of congestion inside, squamous and dry skin, and darkness of the eye sockets” of *On Pulse, Symptom Complex and Treatment of Arthralgia Due to Stagnation of Blood and Consumptive Diseases of Jingui Yaolue* and the sentence “in case of abdominal pain in puerpera, the treatment method should be orange fruit & paeonia powder, and if it is not cured, there should be abdominal congestion below umbilical region” of *On Pulse, Symptom Complex and Treatment of Postpartum Diseases of Jingui Yaolue.* The meaning of congestion can be concluded from the previous opinions as follows:
  1. To become congested means that the state of part of the body being blocked with blood or mucus, and patients with congestion means that they have old blood and blood stasis because of lacking nourishment of qi, blood, and fluid.
  2. The main causes of congestion include improper diet, distress, improper drinking, excessive sexual intercourse, damage due to hunger, or overstrain injury that results in injured meridian, nutrient qi, and defensive qi and then forms stagnation of blood. With internal stagnation and intermingling of blood stasis, failure to neovascularization, and removing old blood, congestion is formed, which was discussed similarly in *Theory of Blood Syndrome* [27].
  3. The nature of congestion is the “bad blood” or “dead blood” that lacks normal nourishment and metabolic function for neovascularization.
  4. The diseases of congestion are divided into the congestion disease and consumptive congestion disease, with essential differences. The congestion disease is the coagulation of congestion and static blood and poison, with shorter course, mild condition, remained vital qi, and shallow and small accumulation of congestion, better treatment effect, and prognosis, which can be treated with the Xiayuxue decoction formula. While the consumptive congestion disease is formed from long-term congestion disease that results in endogenous cancer toxicity and accumulative abdominal mass, leading to extremely weak viscera and primordial qi and deficient and declined qi and blood, with the manifestations of squamous and dry skin and darkness of the eye sockets without blood nourishment. Its condition is severe and the treatment effect and prognosis are poor.
(II) “Extreme weakness due to five consumptions leads to emaciation and abdominal distension with no ability to eat” and describes the “incurable disease” in TCM, as well as the manifestation of late cancer. In *Suwen: Xuanming Five Qi*, it was pointed out that “Long-term viewing injuries the blood, long-term lying injuries the qi, long-term sitting injuries the flesh, long-term standing injuries the bones, and long-term walking injuries the tendons, and together, they are called the injuries by five consumptions.” In *Suwen: Yuji Zhenzang Lun*, “Huangdi asked: I heard that both excess and deficiency are life-threatening, can you introduce it in detail? Qibo said: Five-excess and five-deficiency can cause death. Huangdi asked: Could you tell me what are five-excess and five-deficiency? Qibo said: The five-excess contains five symptoms including vibrant pulse, skin fever, abdominal bloating, obstruction of urine and stool, and delirium, and five-deficiency contains five symptoms including fine pulse, cold skin, less qi, incontinence of urine and stool, and incompatibility of diet” [28]. Ancient annotators Wang Bing said: “Five-excess and five-deficiency come from the five viscera” [29]. Zhang Jingyue believed that “five-excess and five-deficiency originate from the five viscera, and either five-excess or five-deficiency can lead to death” and that “Naturally, complete deficiency of vital energy is incurable” [30]. Long-term “injuries by five consumptions” results in “five-deficiency;” “emaciation” is the external manifestation of “extreme weakness,” “abdominal distension” is the symptom of “abdominal bloating and obstruction of urine and stool” of “five-excess,” “no ability to eat” refers to “incompatibility of diet,” and “less qi” is one of the symptoms of “five-deficiency.” “Abdominal distention” used in the original text shows that patients have obviously distended abdomen, hard mass or tympanites which can be felt by pressing, or accumulation, mass, or ascites which can be confirmed by touching, causing obstruction of urine and stool, severe congested ascending or descending movement of vital qi, and inability of eating and digesting, with the disease location mainly at the middle and lower jiao. If the qi and blood generated by the acquired essence from food and drink have dried up, there is no nourishment provided for the five internal organs, qi, blood, flesh, bones, and tendons; extreme weakness and emaciation due to five consumptions will occur. It is the clinical expression of incurable disease of “five-excess and five-deficiency” in *Huangdineijing* and the clinical inheritance and development of viscera theory in *Huangdineijing* by Zhang Zhongjing. In Zhang Tianxing's opinion, “five-excess” is qi movement congesting (block pattern), and “five-deficiency” is deficient original qi (collapse pattern). The clinical manifestation of five-excess and five-deficiency is respectively the sign of constrain and scattering [31], indicating late cancer, which should be treated by principles of reinforcement and elimination in combination and relaxing spleen-stomach and restoring vital energy.
(III) “Improper diet, distress, improper drinking, excessive sexual intercourse, damage due to hunger, or overstrain injury that results in injured meridian, nutrient qi, and defensive qi” is the important cause and pathogenesis of “congestion,” “congestion disease,” and cancer. There are two levels of meaning. Immoderate diet, malnutrition, excessive drinking, fleshliness, internal injuries caused by seven emotions, strain injury, and damage to meridian, qi, blood, bones, tendons, and defensive qi due to blocked stasis caused by exogenous pathogen invading fleshy exterior which can get worse and then cause extreme consumption of five viscera, leading to the consumed essence, blood, and fluid and then forming the congestion disease. Ancient annotator Xu Zhongke said “Five consumptions mean deficiency in blood, qi, flesh, bone, and tendon.” “In terms of the cause of the disease, it can be their diet, emotion, sexual intercourse, hunger, consumption, and disharmonious meridian, nutrient qi, and defensive qi, which can progress to the extreme. If internal congestion is formed and not removed, the disease cannot be cured.” On the contrary, long-term “internal congestion” can develop into “extreme weakness due to five consumptions, which leads to emaciation and abdominal distension with no ability to eat,” and “squamous and dry skin and darkness of the eye sockets” are the severe symptoms of consumptive congestion disease. The author believed that many noncancerous chronic lesions in modern medicine, such as uterus myoma and endometrial hyperplasia, as well as various benign tumors and polyps, chronic fibroproliferative changes in tissues, and atheromatous lesions of the heart and brain vessels, can be treated based on syndrome differentiation of the theory of congestion disease, and the principle of treatment should be focusing on removing toxicities and supplementing with vital energy restoration.
(IV) The formula of DHZCP presents the treatment principles of reinforcement and elimination in combination and relaxing spleen-stomach and restoring vital energy. The main herbs in the Xiayuxue decoction formula for congestion disease, including cooked rhubarb, ground beetle, and peach seed, as well as multiple herbs such as white grub, gadfly, and leech, are used as the sovereign drug, to soothe and relax the distended abdomen (one of the symptoms of five-excess), strongly remove the extravasated blood, accumulated blood stasis, abdominal mass, and retained food and drink, purge the stomach, promote the metabolism function, facilitate urine and feces excretion, and relieve the pathogenic qi, thereby eliminating various toxicities and abdominal distention, stabilizing and harmonizing five viscera, promoting the ascending or descending movement of vital qi, and quickly exerting the effects of relieving, smoothing, and stabilizing the stomach-spleen. Liquorice root, Chinese peony, adhesive rehmannia dried root, dried lacquer, Baikal skullcap root, and bitter apricot seed are used as the minister drug, mainly to tonify spleen for nourishing qi, replenish essence, and supplement the blood, eliminate hot and cold blood bi and various toxicities, and consolidate stomach-spleen, and nourish the spleen and kidney. The sovereign drug and minister drug are made into pills with honey, so as to persistently and continuously exert the effects of nourishing qi, tonifying spleen and stomach, relieving pain, stabilizing the five-deficiency of viscera, curing the pathogenic qi, and eliminating various toxicities. The pills should be orally taken with Chinese rice wine, which has pungent, warm, sweet, and bitter property and nature, to warm yang and nourish qi, promote qi to activate blood, activate meridians and collaterals, and nourish blood to promote angiogenesis, so that all herbs can work deeply in human body and straight to the lesion location. The formula treats both excess and deficiency, combines reinforcement with elimination, eliminate the pathogenic qi without damaging the vital qi, which is a classic formula in the treatment of “congestion,” “congestion disease,” and “consumptive congestion disease.” Using this theory to guide clinical syndrome differentiation and treatment and modifying the dosage and usage can play an important role in TCM preventive treatment of cancers, early, middle, and late treatment and clinical prevention of other chronic diseases.

## Figures and Tables

**Figure 1:** Between-group comparison of mental status after treatment [Mean ± SD]. Note: the horizontal axis indicated groups B and A, and the vertical axis indicated the HAMA score (points). After treatment, the mean HAMA score of groups B and A was, respectively, (15.61 ± 1.44) and (18.67 ± 1.31); ^*∗*^indicated significant between-group difference in mean HAMA score after treatment (*t* = 11.003 and *P* < 0.001).

**Table 1:** Between-group comparison of clinical data (*n* = 49).

Item	Group A	Group B	*X* ^2^/*t*	*P*
Mean age (Mean ± SD, years)	61.04 ± 3.86	60.57 ± 3.82	0.683	0.496
Mean course of disease (Mean ± SD, months)	27.42 ± 2.66	26.87 ± 2.31	1.093	0.277
Gleason score (Mean ± SD, points)	4.12 ± 0.99	4.22 ± 1.16	0.459	0.647
KPS score (Mean ± SD, points)	78.47 ± 4.06	78.31 ± 3.71	0.204	0.839
Pathological type				
Cystadenocarcinoma	43 (87.76%)	45 (91.84%)	0.446	0.505
Squamous cell carcinoma	1 (2.04%)	2 (4.08%)	0.344	0.558
Neuroendocrine carcinoma	5 (10.20%)	2 (4.08%)	1.385	0.239
Tumor stage			0.176	0.675
Early	32 (65.31%)	30 (61.22%)		
Mid-term	17 (34.69%)	19 (38.78%)		
Educational degree				
College	2 (4.08%)	5 (10.20%)	1.385	0.239
High school	21 (42.86%)	22 (44.90%)	0.041	0.839
Primary school	26 (53.06%)	22 (44.90%)	0.653	0.419
Place of residence			0.165	0.685
Urban area	21 (42.86%)	23 (46.94%)		
Rural area	28 (57.14%)	26 (53.06%)		

**Table 2:** Between-group comparison of complication treatment effect within 3 months (*n* (%)).

Group	*n*	Urinary irritation syndrome	Abnormal defecation	Anal, rectal, and perineal tenesmus, swelling, and pain	Total effective rate
A	49	0	0	0	0
B	49	4 (8.16)	2 (4.08)	3 (6.12)	18.37 (9/49)
*X* ^2^					9.910
*P*					<0.05

**Table 3:** Between-group comparison of complication treatment effect within 3–4 months (*n* (%)).

Group	*n*	Urinary irritation syndrome	Abnormal defecation	Anal, rectal, and perineal tenesmus, swelling, and pain	Total effective rate
A	49	3 (6.12)	2 (4.08)	3 (6.12)	16.33 (8/49)
B	49	9 (18.37)	10 (20.41)	8 (16.33)	55.10 (27/49)
*X* ^2^					16.044
*P*					<0.001

**Table 4:** Between-group comparison of complication treatment effect within 4–6 months (*n* (%)).

Group	*n*	Urinary irritation syndrome	Abnormal defecation	Anal, rectal, and perineal tenesmus, swelling, and pain	Total effective rate
A	49	5 (10.20)	4 (8.16)	4 (8.16)	26.53 (13/49)
B	49	19 (38.78)	13 (26.53)	11 (22.45)	87.76 (43/49)
*X* ^2^					37.500
*P*					<0.001

**Table 5:** Between-group comparison of biological recurrence status during follow-up (*n* (%)).

Item	Group A (*n* = 49)	Group B (*n* = 49)	*X* ^2^	*P*
Biological recurrence/months				
0–30	0	0		
31–48	1 (2.04)	0		
49–60	3 (6.12)	1 (2.04)		
Total	4 (8.16)	1 (2.04)	1.897	0.168
Clinical recurrence/months				
0–30	0	0		
31–48	0	0		
49–60	3 (6.12)	0		
Total	3 (6.12)	0	3.095	0.079

## Data Availability

The data used to support the findings of this study are available from the corresponding author upon reasonable request.
